# Identifying leaks in the STEM recruitment pipeline among sexual and gender minority US secondary students

**DOI:** 10.1371/journal.pone.0268769

**Published:** 2022-06-03

**Authors:** Casey D. Xavier Hall, Christine V. Wood, Manuel Hurtado, David A. Moskowitz, Christina Dyar, Brian Mustanski

**Affiliations:** 1 Institute for Sexual and Gender Minority Health and Wellbeing, Northwestern University, Chicago, IL, United States of America; 2 Department of Medical Social Sciences, Northwestern University, Chicago, IL, United States of America; 3 Department of Public Health Sciences, The University of Chicago, Chicago, IL, United States of America; 4 College of Nursing, Ohio State University, Columbus, OH, United States of America; University of Texas Southwestern Medical Center at Dallas, UNITED STATES

## Abstract

**Purpose:**

Research establishes the critical need to address the underrepresentation of women and racial/ethnic minorities in science, technology, engineering, and mathematics (STEM). While emergent research addresses similar challenges for sexual and gender minorities (SGM), this research remains scant and focuses on adult experiences. This analysis examines subgroup differences and the impact of bullying on STEM engagement outcomes among a national sample of SGM secondary students in the U.S.

**Method:**

This report provides descriptive and multivariable regression analysis of national survey data (n = 539) on the experiences of pre-college students who identify as SGM, including the effects of within-school anti-SGM bullying on STEM identity, perceptions of STEM climate, and STEM intentions.

**Results:**

Roughly 50% of the sample intended to enter a STEM field (compared to 25% in previous general samples). Bullying in school was negatively associated with STEM identity and perceptions of STEM climate. Sense of belonging is positively associated with perceptions of STEM climate and STEM intentions. Being non-binary and being a transgender man were associated with decreased sense of belonging and negative perception of STEM climate.

**Conclusion:**

This report is the first to identify factors influencing STEM engagement among SGM secondary students and suggests that issues of STEM engagement are already present in adolescence. Moreover, the findings also establish the relationship between anti-SGM bullying and STEM outcomes highlighting the importance of this marginalization experience. Future research should further examine sub-group differences and the persistence of these effects. These findings highlight the need for research and intervention addressing STEM outcomes in SGM populations.

**Clinical trial registration:**

https://clinicaltrials.gov/ct2/show/NCT03511131.

## Introduction

Over the past several decades, a great deal of federal funding and person-power have been committed to diversifying the science, technology, engineering, and math (STEM) pipelines, with mixed results. The “diversity dilemma,” as it is aptly known [1], has focused almost exclusively on low rates of participation among women and members of historically underrepresented racial and ethnic groups (“UR,” which includes Black/African American, Latino/a, Pacific Islander, Alaska Native, and Native American scientists). Recently, the National Science Foundation and the National Institutes of Health (NSF and NIH, respectively) have also collected data on and directed support for persons with disabilities in science [2]. These efforts have not included or emphasized sexual and gender minorities (SGM), a population whose experiences and specific needs have been largely overlooked in the research on STEM diversity.

Although recent efforts to examine the experiences of minoritized individuals have not emphasized SGM, they demonstrate the STEM diversity dilemma persists for women and UR individuals. Adapting the definition used by Gillborn 2005, the term ‘minoritized’ refers to the resulting relative status of groups that are often labeled “minority” (e.g., racial-ethnic groups and women) through exclusionary and violent practices of groups with more societal power [3]. This term highlights that this status may exist regardless of numeric minority status. Rather, it is a result of historical and contemporary forms of systemic disadvantage. The research collected on the experiences of women and UR individuals have consistently demonstrated that members of these groups experience more adversity than their well-represented counterparts at all stages of training, mentoring, and career progression, and that their interest in scientific research careers declines early and at disproportionately high rates [4,5]. For example, while the participation of women and UR individuals in biomedicine is improving at faster rates than for other STEM disciplines, their representation remains stagnant at the highest levels of the scientific workforce. Women comprise only 33% of tenure-track research faculty in biomedicine (despite comprising more than 50% of the graduate student population in these fields) and Black/African American scientists represent an astoundingly low proportion of biomedical faculty. Participation rates of women and URs are lower across other STEM fields, particularly engineering, physics, and more mathematics-oriented sciences [2]. While the literature addressing the representation of women and UR individuals is well established, research addressing SGM populations as minoritized scientists is an emergent body of work and remains nascent.

### Sexual and gender minorities (SGM) are an overlooked category

Very little is known about the experiences of SGM scientists across STEM fields. The category of SGM is broad, but in common usage includes lesbian, gay, bisexual, transgender, queer, and intersexed people (LGBTQI). Currently, the National Science Foundation (NSF) does not collect or report data on sexual identity in its various surveys of Science and Engineering fields, including the National Survey of College Graduates, Survey of Earned Doctorates, and Survey of Graduate and Postdoctorates in Science and Engineering [2,6]. While the National Institutes of Health (NIH) identified SGM as a health disparity population for research purposes in 2016 [7], SGMs are not included in the categorization of minoritized individuals within the science education and career pipelines. While the recognition of SGM health disparities is important, NIH positions members of SGM communities as the subjects of science, and not as agents or practitioners of science. As a result, little is known about the experiences of SGM scientists, and this population is not yet recognized in the allocation of federal funds for programs to support and diversify the biomedical and STEM workforces.

Because so little is known about SGMs’ aspiration toward degrees and careers in STEM, serious analysis is needed to understand their experiences at all stages of the pipeline. To begin to understand the potential barriers SGM individuals face when pursuing STEM education and training, original research must explore the experiences of SGM students within STEM learning settings beginning in the elementary or secondary school levels. Indeed, research on gender and racial diversity in STEM has emphasized the importance of creating comprehensive “pathway” practices in elementary and secondary schools, including mentoring and internships, to support UR students throughout the education and training trajectories [8]. Research shows fostering diverse learning environments helps promote retention at all stages of the education and training process and may help mitigate the impacts on how UR students perceive their own abilities based on societal messaging around race and gender [9,10]. This, and other research, also shows UR students in secondary school take fewer courses in math-oriented fields and need additional support for sustaining confidence and interest in these areas [9,11,12]. Further research underscores how supporting aspiring scientists through mentorship and hands-on research experiences early in their education trajectories promotes retention in STEM for women and UR students [13].

Following the abundant research on gender and racial/ethnic underrepresentation in STEM, a sustained examination of the experiences of SGMs will augment the research on young people who aspire to further their education in STEM fields and the barriers they may face. A broad base of robust research on SGM students’ experiences will help in the development of strategies to fortify the pipeline for supporting and retaining aspiring SGM scientists. This report considers the experiences of secondary-school students who identify as SGM and have indicated interest in pursuing STEM coursework and/or careers in the future.

### A paucity of research on SGM STEM experiences

Research estimating the proportion of aspiring scientists who identify as SGM remains scant. Results of one nationally distributed survey for first-year college students (“The Freshman Survey”) found that among 4,325 students who provided data on their sexual and gender identities and academic intentions, 11.9% of those intending to pursue STEM identified as SGM (n = 515) [14]. While this rate is higher than the percentage of individuals from the general US population who choose to disclose their LGBTQI status in national surveys, which has hovered around 4.5% for many years [15], it is similar to or less than the proportion of estimates focusing on Millennial (10.5%) and Gen Z (20.8%) age cohorts, which would be closer age-matched to the Freshman Survey [16]. Thus, it is difficult to draw conclusions about the proportion of scientists who identify as SGM relative to the general population given available evidence. Regardless, understanding SGM students’ experiences as aspiring members of the STEM workforce is an important contribution to the literature on STEM pipeline disparities.

The limited research that does exist on climate issues suggests that SGMs’ experiences within the STEM pipeline are not positive. In a large dataset (n = 4,162) of students across 78 higher education institutions, SGM-identified students aspiring to STEM majors were 9.5% less likely than their heterosexual and/or cisgender counterparts to remain in science by the end of their fourth year of college, despite being more likely to pursue research experiences as part of their studies [17]. In a qualitative study of SGM engineering students, participants described having strong engineering identities, but also described a relative silence around SGM identities in the sciences and concerns about potential discrimination in their future careers [18]. Their concerns are justified; SGM employees working in STEM fields within federal agencies report poorer treatment and lower satisfaction than non-SGM employees. Alarmingly, SGM individuals face some of the highest levels of harassment among NIH employees [19,20]. Other research points to educational climate issues affecting SGMs. This patchwork of research paints an alarming picture of SGM experiences in STEM, beginning early in the educational pipeline and into career stages.

The theoretical basis of this research is the literature on science identity, which spans the fields of psychology and qualitative education research [21,22]. The concept of science identity is broad and refers generally to how people define themselves and self-present as scientists. Much of the research on science identity focuses on undergraduate or graduate students who have decided to pursue STEM education. For example, research on women of color in undergraduate and graduate biology programs has described how adverse experiences in STEM training environments interfere with students’ science identities. This research demonstrates that a person’s science identity and pursuit of success are “disrupted by the interaction with gendered, ethnic, and racial factors" [21]. Thus, the components of science identity important to this paper are experiences of adversity (i.e., anti-SGM bullying) and their association with sense of belonging in STEM learning environments and perceptions of STEM climate. Although this paper does not utilize formal measures for science identity, in part because the subjects of our research do not yet have hands-on experience in STEM training environments, it explores factors known to have negative effects on retention of minoritized individuals. As such, this report serves as an entrée into the relationship between adversity and perceptions of and intentions towards science education.

Social marginalization often referred to as minority stress in the context of SGM populations is a well-established factor in the health and quality of life in SGM populations [23–25]. While some models conceptualizing bully and harassment as a climate issue [26], the literature on minority stress has conceptualized this specific form of social marginalization as operating on multiple levels of the social ecology and multi-faceted such as direct experience of discrimination, anticipated discrimination, and internalized discrimination [23–25]. Social marginalization, which includes bullying, harassment, or lack of support from peers and mentors based on sexual/gender identity, has been identified as a potential barrier to retention in STEM for SGM individuals. Among adult SGM professionals in STEM fields, social marginalization may take the form of workplace harassment and other forms of exclusion or lack of recognition [27]. The logical analogue among young people in the context of secondary school is anti-SGM bullying, which may be conceptualized as a precursor to other SGM-specific marginalization experiences in college and the workforce.

Although point estimates vary, prevalence of bullying among SGM youth has been 50% or higher in some studies, including school-based and cyber bullying [28,29]. Anti-SGM bullying has been linked to a variety of negative outcomes among SGM adolescents, including depression, anxiety, substance abuse, low self-esteem, and suicide [28]. While no known studies have examined the effects of bullying on STEM pipeline outcomes for SGM students, general research on bullying victimization has been linked to negative educational outcomes, including reduced school belonging, academic disengagement, reduced academic aspirations, and poor academic performance [28]. Many of these academic outcomes could preclude or disadvantage an individual from entering or persisting in the highly competitive world of STEM careers.

While these findings describe the consequences of social marginalization on the overall academic performance and well-being of SGM adolescents, they do not speak directly to the impacts of adolescent experiences of social marginalization. Nor do they fully address anti-SGM bullying as a potentially influential determinant of STEM engagement situated within the life-course of would-be STEM professionals. Rather, this report is the first of its kind to examine the experiences of pre-college students who identify as SGM and demonstrate interest in continuing in STEM as they further their education. More specifically, this report addresses these questions:

- Are there differences in STEM intent across fields by gender, sex assigned at birth and sexual identity?
- Is anti-SGM bullying related to sense of belonging in STEM classes and perceptions of classroom climate among pre-college students?
- Are sense of belonging and perceptions of STEM climate associated with STEM intent in SGM students?

## Method

### Study design and recruitment

Data for this cross-sectional study were collected between July 2019 and July 2020 primarily through social media advertising, which promoted participation in an ongoing HIV prevention trial. More details on this trial have been described elsewhere [30]. Those that did not meet the eligibility requirements for that ongoing study were redirected to a separate survey focusing on STEM perceptions. To be eligible for this study, participants had to be between 13–18 years old and live in the U.S. Eligible participants completed an online consent form. Upon survey completion, participants were entered into a raffle to win one of twenty $25 gift cards. All these procedures were approved by Northwestern Institutional Review Board (STU00201997) with waivers of parental permission [31].

#### Description of sample

There was a total of 539 participants. All participants provided data on all measures used in this study. Table 1 presents a descriptive summary of the sample. Almost half (*n* = 266; 49.35%) of participants indicated an intent to enroll in a STEM field. The sample reported, on average, that they experienced some degree of bullying, with few (*n* = 5; >1.0%) participants indicating that they were never bullied because of their sexual or gender identity at school in the past year. Participants were also asked about sense of belonging in STEM learning environments, or how they felt in math or science class. Participants generally reported a neutral sense of belonging in math class and in science class, meaning that they did not particularly feel thrilled or miserable in those classes. Similarly, perceived STEM climate of LGBQ people and for transgender people were also distributed normally around a neutral score (approximately five out of ten).

**Table 1:** Description of the sample of sexual and gender minority secondary school students in the U.S. (n = 539).

		Count	%	
Age (categorical)	13	19	3.53	
	14	51	9.46	
	15	105	19.48	
	16	135	25.05	
	17	160	29.68	
Gender Identity	18 Cisgender men	69 292	12.80 54.17	
	Transgender men Non-binary	191 34	35.44 6.31	
Sexual Identity	Cisgender & Transgender women Gay/Lesbian	22 276	4.08 51.21	
	Bisexual	135	25.05	
	Pansexual	55	10.20	
	Queer	36	6.68	
Race/Ethnicity	Unsure/Questioning or other sexual identity	37	6.86	
	White	307	57.00	
	Latinx/Hispanic	119	20.22	
	Black/African American	25	9.83	
	Asian	35	8.72	
	AI/NA/NH/OPI	7	4.08	
	Multiracial	46	8.5	
STEM Intent		266	49.35	
*Unless noted*, *N = 539*		Skew (SE)	Kurtosis (SE)	Range
Age		-.44 (.11)	-.52 (.21)	13.08–18.84
Bullying Affective Experiences Sense of belonging in math class		.37(.11) -.24 (.11)	-.11(.21) -.85 (.21)	1–5 1–10
Sense of belonging in science class		-.46 (.11)	-.61 (.21)	1–10
Perceived STEM Climate How welcoming people in STEM fields are of LGBQ people		.13 (.11)	-.63 (.21)	1–10
How welcoming people in STEM fields are of transgender people		.60 (.11)	-.34 (.21)	1–10

### Measures

#### Anti-SGM bullying

Marginalization experiences were conceptualized as anti-SGM bullying in the school setting. A 10-item measure was used to assess SGM-related experiences of bullying in school in the past year [32]. Each question-item (e.g., “In the past year, how often have you been physically assaulted at your school because you are LGBTQ?”) was rated on a 5-point scale (1 = never, 5 = frequently), and averaged to create a total score (α = .86).

#### Sense of belonging in STEM learning environments

Sense of belonging in STEM learning environments was operationalized using the Institutional Belonging Scale by more broadly adapting it to assess the level of belonging students felt in math and science classes [33]. This measure has been shown to measure African American college student’s sense of belonging in the university (α = .92). Findings showed that participants with higher sensitivity to race-based rejection reported a significantly lower sense of belonging. For the current analysis, four question-items were developed for each type of class (e.g., “Think about how you feel in math class, how thrilled/excited are you in the class?”), rated on a 10-point scale (1 = miserable to be there, 10 = very thrilled), and averaged to create two scores: one for math (α = .90) and one for science (α = .91).

#### Perceived STEM climate

Perceived STEM climate was operationalized using adapted items from the college campus climate study [34]. In this case SGM identities were separated into two categories: 1) lesbian, gay, bisexual, queer (LGBQ), and 2) transgender. One item was used for each identity group to measure participant perceptions of the extent to which people in STEM fields are welcoming to the specific identity group listed (either LGBQ or transgender). For example, the question regarding LGBQ individuals read: “How welcoming do you think people in STEM fields are of LGBQ people?” The degree of welcome was then assessed on a 10-point scale (1 = not at all welcoming, 10 = very welcoming).

#### STEM intent

Participants were asked to select all the fields of study that they intended to enroll in. These individual fields were used in an exploratory bivariate analysis (see Table 2). We then created a dichotomous variable to indicate interest in enrolling in a STEM field (computer/information science, engineering, life sciences, mathematics, medical sciences, or physical sciences).

**Table 2:** Exploratory bivariate analyses of intended college field of study by gender identity and sexual identity.

	**STEM Fields**											
	Computer, Information Science		Engineering		Life Sciences		Mathematics		Medical Sciences		Physical Sciences	
	n, (%)	Sig.	n, (%)	Sig.	n, (%)	Sig.	n, (%)	Sig.	n, (%)	Sig.	n, (%)	Sig.
Gender Identity^a^												
Cisgender & Transgender women	2 (9.1%)	0.072^b^	4 (18.2%)	0.012^b^**	2 (9.1%)	.841^b^	2 (9.1%)	.012^b^**	3 (13.6%)	.255^b^	3 (13.6%)	.406^b^
Non-binary Transgender men	5 (14.7%) 13 (6.8%)		2 (5.9%) 9 (4.7%)		5 (14.7%) 25 (13.1%)		4 (11.8%) 4 (2.1%)		3 (8.8%) 31 (16.2%)		3 (8.8%) 14 (7.3%)	
Cisgender men Sexual Identity^a^ Unsure/Questioning or other	48 (16.4%) 6 (16.2%)	0.843^b^	43 (14.7%) 6 (16.2%)	.182^b^	47 (16.1%) 2 (5.4%)	.414	36 (12.3%) 4 (10.8%)	.182^b^	68 (23.3%) 4 (10.8%)	.414	38 (13.0%) 6 (16.2%)	.573^b^
sexual identity												
Queer	3 (8.3%)		0 (0%)		6 (16.7%)		5 (13.9%)		5 (13.9%)		1 (2.8%)	
Pansexual	5 (9.1%)		3 (5.5%)		5 (9.1%)		11 (20.0%)		11 (20.0%)		5 (9.1%)	
Bisexual	17 (12.6%)		18 (13.3%)		19 (14.1%)		22 (16.3%)		22 (16.3%)		15 (11.1%)	
Gay/Lesbian	37 (13.4%)		31 (11.2%)		47 (17.0%)		63 (22.8%)		63 (22.8%)		31 (11.2%)	
	**Other Fields**											
	Art		Business		Education		Humanities		Journalism, Communications		Social Sciences	
	n, (%)	Sig.	n, (%)	Sig.	n, (%)	Sig.	n, (%)	Sig.	n, (%)	Sig.	n, (%)	Sig.
Gender Identity^a^												
Cisgender & Transgender women	1 (4.5%)	0.696^b^	1 (4.5%)	0.048^b^**	3 (13.6%)	.553^b^	4 (18.2%)	.391	1 (4.5%)	.341^b^	4 (18.2%)	.532
Non-binary Transgender men	4 (11.8%) 28 (14.7%)		4 (11.8%) 12 (6.3%)		7 (20.6%) 22 (11.5%)		10 (29.4%) 57 (29.8%)		6 (17.6%) 21 (11.0%)		12 (35.3%) 61 (31.9%)	
Cisgender men Sexual Identity^a^ Unsure/Questioning or other	34 (11.6%) 4 (10.8%)	0.977^b^	47 (16.1%) 4 (10.8%)	.678^b^	32 (11.0%) 6 (16.2%)	.779^b^	63 (21.6%) 10 (27.0%)	.414	21 (7.2%) 8 (21.6%)	.178^b^	79 (27.1%) 11 (29.7%)	.406
sexual identity												
Queer	5 (13.9%)		4 (11.1%)		6 (16.7%)		14 (38.9%)		6 (16.7%)		16 (44.4%)	
Pansexual	7 (12.7%)		6 (10.9%)		7 (12.7%)		15 (27.3%)		4 (7.3%)		19 (34.5%)	
Bisexual	15 (11.1%)		11 (8.1%)		14 (10.4%)		35 (25.9%)		11 (8.1%)		36 (26.7%)	
Gay/Lesbian	36 (13.0%)		39 (14.1%)		31 (11.2%)		60 (21.7%)		20 (7.2%)		74 (26.8%)	

^a^n may vary.

^b^Fisher’s Exact Test.

* p < .05

** p < .01

*** p < .001.

#### Demographic characteristics

Participants reported their birthdates (used to calculate age), their sex assigned at birth (male, female, or intersex) and gender identity (male, female, transgender, non-binary, genderqueer/gender non-conforming, or other). These items were part of the parent study on HIV and follow guidance for assessing transgender identity from lead transgender health researchers [35]. Sex assigned at birth and gender identity were collapsed into a single variable, which included “cisgender man,” “woman,” “transgender man,” and “non-binary” (non-binary, gender non-conforming or other gender identities). The “cisgender woman” and “transgender woman” categories were combined into a single woman category due to limited representation in this sample. Participants self-reported their sexual identity, which was also recoded due to limited representation of certain identities into the following: gay/lesbian, bisexual, pansexual, queer, and unsure/questioning or other identity. Similarly, participant’s race/ethnicity data were recoded into the following groups: White, Latinx/Hispanic, Asian, Black or African American, American Indian/Native Alaskan/Native Hawaiian/Other Pacific Islander (AI/NA/NH/OPI), or multi-racial.

### Analytic plan

Data were analyzed using SPSS 27, and all 539 participants provided data on all measures used in this study. Descriptive statistics were calculated and used to assess assumptions for planned tests (e.g. normality). A confirmatory factor analysis based on eigenvalues, using maximum likelihood extraction and direct oblimin rotation was conducted to assess both of the adapted sense of belonging in STEM learning environments scales. A series of Pearson correlations were conducted to examine associations among bullying, sense of belonging in STEM learning environments, perceived STEM climate, and STEM intent. An exploratory bivariate analysis (Chi-square test of independence, and Fisher’s exact test) was conducted to examine the distribution of sexual identities, and gender identities in each intended field of study. Simple logistic regression analyses were employed to assess the relationships among demographic characteristics, bullying, sense of belonging in STEM learning environments, perceived STEM climate, and STEM intent. Following those analyses, multiple regressions were employed to generate adjusted estimates of effects on sense of belonging in STEM learning environments, perceived STEM climate, and STEM intent. Standardized beta coefficients, standard errors, and adjusted odds ratio (aOR), and 95% confidence intervals are reported accordingly. We also investigated outliers in bullying, sense of belonging in STEM learning environments, and perceived STEM climate using the interquartile range method. There was only one outlier case found within STEM bullying. We conducted sensitivity analyses excluding this case and found no differences in our results. Our approach to dealing with Type-I error rate inflation due to multiple comparisons included employing an alpha correction that adjusted the false discovery rate using the Benjamini-Hochberg procedure, and we report the corrected significance levels [36]. G*Power [37] was used to perform an a priori power analyses for linear and logistic regression analyses to determine a sufficient sample size. For small to medium effect sizes (.20 or greater) among planned linear regression analyses and a minimum odds ratio detection of 1.5 among logistic regression analyses, our analyses are well-powered (power = .99; α = .05) given our sample sizes.

#### Confirmatory factor analysis

The factor structure of the four question-items comprising each of the sense of belonging in STEM learning environments scales were examined. Initial eigenvalues indicated that Factor 1, comprised of 4 items assessing sense of belonging in math class, explained 76.97% of the variance with factor loadings ranging from .720 to .926. A one factor solution was preferred because of its previous theoretical support, and the scree plot and eigenvalues ‘leveled off’ after one factor. Similarly, initial eigenvalues indicated that the single factor, comprised of four items assessing sense of belonging in science class, explained 78.40% of the variance with factor loadings ranging from .750 to .918. Likewise, a one factor solution was preferred because of its previous theoretical support, and the eigenvalues and scree plot ‘leveled off’ after one factor. Overall, this exploratory factor analysis indicated that one distinct factor explained SGM adolescent responses to each of the sense of belonging in STEM learning environments scales, and that both factors displayed excellent internal consistency.

## Results

### Exploratory descriptive analysis of intended fields of study

Table 2 presents the chi-square analyses used to determine the bivariate associations between fields of interest (sorted STEM and non-STEM) and demographic characteristics (gender identity and sexual identity). In our sample, the associations between gender identity and the following intended fields of study were significant: computer/information science, engineering, mathematics, and business. Cisgender and transgender women were most likely to be interested in engineering followed by cisgender men, non-binary participants, and then transgender men. Cisgender men were most likely to be interested in mathematics followed by non-binary participants, cisgender and transgender women, and then transgender men. Cisgender men were most likely to be interested in business followed by non-binary participants, transgender men, and then cisgender and transgender women. There were no significant associations between sexual identity and intended field of study.

### Examining associations with sense of belonging in STEM learning environments and perceived STEM climate

A correlation matrix is presented in Table 3. There was a statistically significant, negative relationship between participant’s age, and bullying, and participant’s perceptions of how welcoming people in STEM fields are of transgender people. There was a statistically significant, negative association between bullying, and sense of belonging in STEM learning environments and perceived STEM climate. Sense of belonging in math class was significantly, positively associated with perceptions of science class, perceived STEM climate, and STEM intent. Perceptions of science class was significantly, positively associated with perceived STEM climate and STEM intent. There was a significant, positive association between participant’s perceptions of how welcoming STEM fields are of LGBQ people, and STEM intent and how welcoming people in STEM fields are of transgender people. Finally, there was a significant, positive association between STEM intent, and participant’s perceptions of how welcoming STEM fields are of transgender people.

**Table 3:** Means, standard deviations, and pearson correlations of age, bullying, sense of belonging in STEM learning environments, perceived STEM climate, and STEM intent.

*Variable*	*M*	*SD*	1	2	3	4	5	6	7
1. Age	16.57	1.30	-						
2. Bullying	2.43	0.70	-.18***	-					
3. Sense of belonging in math class	5.98	2.41	-.04	-.34***	-				
4. Sense of belonging in science class	6.90	2.21	.02	-.21***	.47***	-			
5.Welcoming of LGBQ people	5.68	2.21	-.05	-.29***	.33***	.28***	-		
6. Welcoming of transgender people	4.36	2.41	-.10*	-.27***	.29***	.27***	.78 ***	-	
7. STEM intent	0.49	0.50	-.04	-.06	.29***	.28***	.16 ***	.16 ***	-

* p < .05

** p < .01

*** p < .001.

Table 4 presents the adjusted estimates. All four multiple regression models were significant: sense of belonging in math class (F(13,525) = 13.610, p < .001, R^2^ = .252), sense of belonging in science class (F(13,525) = 4.520, p < .001, R^2^ = .101), how welcoming people in STEM fields are of LGBQ identities (F(15,523) = 8.907, p < .001, R^2^ = .203), and how welcoming people in STEM fields are of transgender identities (F(15,523) = 7.832, p < .001, R^2^ = .183). After adjusting for covariates and applying a p-value correction for multiple tests the following observations were made. Cisgender and transgender women had a significantly lower sense of belonging in math class compared to cisgender men. Transgender men had significantly lower sense of belonging in STEM learning environments, and a significantly lower sense of how welcoming people in STEM fields are of LGBQ people. Non-binary students had a significantly lower sense of how welcoming people in STEM fields are of LGBQ people only. Relative to gay/lesbian participants, queer participants reported a significantly lower sense of belonging in math class. Older age was significantly, negatively associated with participant’s sense of belonging in math class and how welcoming people in STEM fields are of transgender people. Relative to white peers, Black participants reported lower sense of how welcoming STEM fields are for LGBQ people. Experiencing bullying was significantly, negatively associated with sense of belonging in STEM learning environments and perceived STEM climate across all four outcomes. Participant’s sense of belonging in math class was positively associated with their perceptions of how welcoming people in STEM fields are of LGBQ people. Finally, participant’s sense of belonging in science class was significantly, positively associated with their perceptions of STEM climate across both outcomes.

**Table 4:** Multiple linear and logistic regressions examining influences on Sense of belonging in STEM learning environments and perceptions of STEM climate.

	Affective Experiences				Perceptions of STEM Climate				
		Sense of belonging in math class		Sense of belonging in science class		Welcoming of LGBQ people		Welcoming of transgender people		STEM Intent
	β_adj_ (SE)	Standardized β_adj_	β_adj_ (SE)	Standardized β_adj_	β_adj_ (SE)	Standardized β_adj_	β_adj_ (SE)	Standardized β_adj_	aOR (95% CI)
Gender Identity (Cisgender men ref.)									
Cisgender & transgender women	-1.24 (0.48)*	-.10	-0.42 (0.49)	-.04	-0.16 (0.47)	-.01	-0.27 (0.51)	-.02	0.76 (0.30–1.96)
Non-binary	-0.82 (0.41)	-.09	-0.84 (0.42)	-.09	-1.25 (0.40)**	-.14	-0.91 (0.43)	-.09	0.88 (0.40–2.03)
Transgender men	-1.23 (0.22)**	-.25	-0.78 (0.22)**	-.17	-0.80 (0.22)**	-.17	-0.54 (0.24)	-.11	0.77 (0.49–1.21)
Sexual Identity (Gay/Lesbian ref.) Unsure/Questioning	-0.62 (0.38)	-.07	0.43 (0.38)	-.05	0.08 (0.37)	.01	0.08 (0.40)	.01	1.15 (0.54–2.45)
or other sexual identity									
Queer	-1.41 (0.39)**	-.15	-0.60 (0.40)	-.07	0.13 (0.39)	.01	-0.14 (0.42)	-.01	0.91 (0.40–2.07)
Pansexual	-0.57 (0.33)	-.07	-0.50 (0.34)	-.07	0.35 (0.32)	.05	0.63 (0.35)	.08	0.86 (0.44–1.70)
Bisexual	-0.25 (0.23)	-.04	0.04 (0.23)	.01	0.20 (0.22)	.04	-0.03 (0.24)	-.01	1.11 (0.70–1.76)
Race/Ethnicity (White ref.) AI/NA/NH/OPI	0.11 (0.82)	.01	-0.53 (0.83)	-.03	0.58 (0.80)	.03	0.72 (0.86)	.03	3.84 (0.62–23.51)
Asian	0.92 (0.38)	.09	0.40 (0.39)	.04	0.09 (0.38)	.03	0.33 (0.40)	.03	2.76 (1.18–6.45)
Black/African-	0.11 (0.45)	.01	0.09 (0.45)	.01	-1.09 (0.43)	-.10*	-0.76 (0.47)	-.07	1.01 (0.41–2.47)
American Latinx/Hispanic	0.39 (0.24)	.07	0.16 (0.24)	.03	0.08 (0.02)	0.02	0.29 (0.24)	.05	0.93 (0.58–1.47)
Multiracial	-0.04 (0.34)	-0.35	0.09 (0.45)	.01	0.12 (0.33)	0.02	-0.24 (0.36)	-.03	1.76 (0.90–3.47)
Age	-0.18 (0.07)*	-.11	-0.03 (0.07)	-.02	-0.15 (0.07)	-.09	-0.25 (0.08)**	-.14	0.99 (0.86–1.14)
Bullying	-0.91 (0.14)**	-.26	-0.48 (0.14)**	-.15	-0.59 (0.14)***	-.18	-0.70 (0.15)**	-.20	1.35 (1.00–1.83)
Sense of Belonging in	-	-	-	-	0.13 (0.05)*	.14	0.09 (0.05)	.09	1.21 (1.10–1.33)*
math class									
Sense of Belonging in	-	-	-	-	0.15 (0.05)**	.14	0.18 (0.05)**	.17	1.20 (1.09–1.32)*
science class									
Welcoming of LGBQ people	-	-	-	-	-	-	-	-	0.98 (0.86–1.12)
Welcoming of transgender people	-	-	-	-	-	-	-	-	1.08 (0.96–1.22)

All the analyses utilized the full sample (*N* = 539). The SE, Standard Error.

* p < .05 after correction

** p < .01 after correction

*** p < .001 after correction.

### Examining associations with STEM intent

Table 4 also presents the adjusted logistic regression analysis. Only participants that had higher levels of sense of belonging in STEM learning environments, were significantly more likely to intend on enrolling in a STEM field.

## Discussion

This is the first analysis to examine barriers to STEM fields among SGM secondary school students, building on a small body of literature highlighting significant barriers to success in STEM fields among SGM scientists and a higher degree of marginalization experiences compared to their non-SGM peers [18–20,27]. Overall, nearly half of participants intended on pursuing a STEM discipline, which is higher than roughly 25% in general samples [38,39]. However, previous research observed that 9.6% fewer SGM will graduate with a STEM degree relative to their non-SGM peers [17]. This analysis indicates that issues related to the STEM pipeline begin early for SGM. In particular, this analysis establishes anti-SGM bullying impacts STEM outcomes among SGM secondary school students, which runs parallel to research addressing the experiences of UR individuals and women [1]. When placed in the context of existing literature, these results suggest that barriers to SGM representation in STEM are pervasive across the pipeline. “Leaks” earlier in the pipeline in secondary school pose risks to persistence in STEM and can diminish the representation of SGM-individuals at later stages of the pipeline.

### Sense of belonging, perceptions of STEM climate and STEM intentions among SGM adolescents

This study was innovative in its use of SGM-specific measures, including perceived acceptance of LGBQ identities and perceived acceptance of transgender identities in STEM classroom settings. It is important to measure SGM-specific experiences within STEM climates to discern these unique experiences. This analysis observed that STEM belonging was associated with perceptions of SGM-specific STEM climate. This finding is important, as it suggests a connection between early classroom experiences and overall perceptions of STEM fields. Moreover, we observed an association with STEM sense of belonging and STEM intentions, which underlines the potential for early consequences of diminished sense of belonging in STEM courses among SGM adolescents. Taken together with existing literature, our findings suggest the possibility of enduring consequences of early perceptions of STEM field and provide additional evidence that the SGM population should be considered within the broader category of underrepresented individuals in STEM, as categorized by NIH and NSF.

### Anti-SGM bullying as a barrier to sense of belonging and perceptions of STEM climate

This analysis establishes anti-SGM bullying in schools as a unique form of social marginalization impacting STEM career identity among SGM adolescents. This analysis observed that anti-SGM bullying is correlated with discomfort in STEM classrooms as well as perceptions of acceptance of SGM people in STEM climates in general. While previous literature has established a high degree of social marginalization among SGM STEM professionals [13,27], these findings differ in that anti-SGM bullying in schools (i.e. not exclusive to STEM contexts) may have a detrimental impact on experiences of the science classroom and development of science identity.

The science identity literature emphasizes “recognition” as one key element of science identity formation. That is, recognition by oneself and by others (such as peers or teachers) as a “science person” is critical to the development of a stable science identity, particularly at the early stages of education and training. Initial self-identification with and persistence in science rely on frequent affirmation from others. This literature also establishes that development and maintenance of science identity may be interrupted by discrimination or signs of prejudice against one’s social group [21]. Similarly, the literature on sense of belonging in education has emphasized “social integration” and peer group connection as critical elements. Social integration and peer group connection may refer to opportunities for racial/ethnic group identification and engagement with peers inside and outside of the classroom. While research in this area has focused on higher education and racial/ethnic marginalization, the ability to form socially affirming connections with students who are similarly identified (in our case, SGM) and share interest in an area of coursework (in our case, math and science) is relevant to our findings [22].

At minimum, experiences of anti-SGM bullying in schools should be considered as a potential barrier to developing positive STEM identity for SGM adolescents. However, future research should also examine the ways in which stigmatization may happen within contexts specific to the STEM pipeline or be perpetrated by others within STEM (such as STEM teachers or classmates), because it is possible that bullying experiences that are more closely linked to the STEM context may have more influence on STEM pipeline related outcomes. Moreover, future research should address other factors beyond bullying that have been studied for women and UR in STEM, such as the examples provided in STEM curriculum (e.g. most scientists portrayed as cisgender heterosexual men) and available mentorship (e.g. most STEM teachers being cisgender heterosexual men).

### Subgroup differences among SGM

This analysis was also innovative in that it examined the potential differences by gender and sexual identity among SGM adolescents, which are generally treated as a homogenous category in existing literature. We observed diminished sense of belonging among queer-identified participants relative to gay/lesbian-identified participants in the model for sense of belonging in math class as well as in bivariate associations with sense of belonging in science class and STEM climate. As individuals who identify as queer often report attractions to more than one gender, like bisexual or pansexual individuals (often referred to as bi+), this result is consistent with literature suggesting that bi+ populations are more at risk for stigma and discrimination resulting in negative mental health outcomes as compared to heterosexual and gay/lesbian peers [40]. We observed a similar pattern for pansexual and bisexual participants in bivariate associations with sense of belonging in math class; however, it is unclear why we would not observe a difference for bisexual individuals in adjusted models as well. Given the lack of preexisting literature examining subgroups this result suggests a clear direction for future research.

Moreover, we observed differences by gender identity. Significant bivariate associations were observed across computer science, engineering, mathematics, and physical sciences, though sample sizes were small. While the pattern was not completely consistent, transgender men had the lowest proportion of intention in all four of these fields and women had one of the lowest proportion of intent in computer science and mathematics. In multi-variable models, non-binary individuals and transgender men consistently reported lower sense of belonging and more negative perception of STEM climate. These findings build on the known problems of underrepresentation of cisgender women in STEM professions, by broadening these findings to women more broadly, non-binary individuals and transgender men. Taken together, these subgroup associations highlight the importance of considering differences across various SGM identities in future examination of STEM-related outcomes with a need for closer examination of bi+ populations, non-binary, and transgender populations.

### Implications for the field

This analysis suggests a need for research and interventions to address STEM outcomes among SGM. Researchers seeking to increase SGM representation in STEM may look to existing interventions aimed at increasing STEM representation among cisgender girls, UR students, though such interventions have had mixed results [34,41,42]. They may also look toward other initiatives aimed at increasing SGM representation in secondary school curriculum [43] and decreasing bullying among SGM students [44]. Moreover, federal agencies that fund research on STEM participation should collect data on SGM demographics, fund relevant projects, and incorporate these data into their assessment of underrepresented populations.

### Limitations

This study had many strengths, including a geographically and racially diverse sample as well as SGM-specific measures. Even so, there are some limitations to consider. First, the sampling is cross-sectional and non-random. This limits the generalizability of the findings and the ability to make assumptions of causality. Second, the measure of anti-SGM bullying, while focused on the school context, was not specific to STEM. Future studies should consider anti-SGM bullying exclusively within STEM environments. Measures could also be expanded to encompass other forms of discrimination and stereotyping, such as adverse experiences with teacher and mentors or feelings of exclusion. Further analysis should also explore both the sexual identity and gender identity dimensions of bullying and how these relate to sex-based discrimination in the context of STEM. While the incorporation of multiple SGM identities in this study is a strength, power to detect smaller effect sizes may be limited due to the sample size. Future studies should employ sampling techniques to maximize the power to detect differences across subgroups within SGM adolescents.

### Conclusion

This is the first study to examine antecedents of SGM representation in STEM fields among adolescents. The findings suggest that issues of belonging, perceived STEM climate, and STEM intention are already present in adolescence. Moreover, the findings also establish the relationship between anti-SGM bullying and STEM outcomes highlighting the importance of this marginalization experience. Future research should further examine sub-group differences and the persistence of these effects. These findings highlight the need for research and intervention addressing STEM outcomes in SGM populations across developmental periods.

## References

[1] WomackVY, WoodCV, HouseSC, QuinnSC, ThomasSB, McGeeR, et al. Culturally aware mentorship: Lasting impacts of a novel intervention on academic administrators and faculty. PloS one. 2020;15(8):e0236983. doi: 10.1371/journal.pone.0236983 32764768PMC7413486

[2] Foundation NS. Women, Minorities, and Persons with Disabilities in Engineering and Science 2019. Available from: https://ncses.nsf.gov/pubs/nsf19304/.

[3] GillbornD. Education policy as an act of white supremacy: Whiteness, critical race theory and education reform. Journal of education policy. 2005;20(4):485–505.

[4] GibbsKDJr, GriffinKA. What do I want to be with my PhD? The roles of personal values and structural dynamics in shaping the career interests of recent biomedical science PhD graduates. CBE—Life Sciences Education. 2013;12(4):711–23. doi: 10.1187/cbe.13-02-0021 24297297PMC3846521

[5] LambertWM, WellsMT, CiprianoMF, SnevaJN, MorrisJA, GolightlyLM. Research Culture: career choices of underrepresented and female postdocs in the biomedical sciences. Elife. 2020;9:e48774. doi: 10.7554/eLife.48774 31898935PMC6977964

[6] Health NIo. Sexual and Gender Minorities Formally Designated as a Health Disparity Population for Research Purposes. 2016.

[7] LanginK. How many scientists are LGBTQ? Federal survey delays frustrate researchers: Scientists call for National Science Foundation’s workforce surveys to tally sexual and gender minorities. ScienceInsider. 2020.

[8] CaldwellL, GarciaR, CagleN. K-12 diversity pathway programs in the E-STEM fields: A review of existing programs and summary of unmet needs. Journal of STEM Education: Innovations and Research. 2018;19(4).

[9] FarindeAA, LewisCW. The underrepresentation of African American female students in STEM fields: Implications for classroom teachers. Online Submission. 2012.

[10] ValantineHA, CollinsFS. National Institutes of Health addresses the science of diversity. Proceedings of the National Academy of Sciences. 2015;112(40):12240–2. doi: 10.1073/pnas.1515612112 26392553PMC4603507

[11] AlhaddabTA, AlnatheerSA, editors. Future scientists: How women’s and minorities’ math self-efficacy and science perception affect their STEM major selection. 2015 IEEE Integrated STEM Education Conference; 2015: IEEE.

[12] HinojosaT, RapaportA, JaciwA, ZacamyJ. Exploring the Foundations of the Future STEM Workforce: K-12 Indicators of Postsecondary STEM Success. REL 2016–122. Regional Educational Laboratory Southwest. 2016.

[13] EstradaM, WoodcockA, HernandezPR, SchultzP. Toward a model of social influence that explains minority student integration into the scientific community. Journal of educational psychology. 2011;103(1):206. doi: 10.1037/a0020743 21552374PMC3087606

[14] CobianK. A Comparison of Intended Biomedical Majors Across Sexual and Gender Identity: A First Look from Freshmen at BUILD Sites. Fact Sheet. Los Angeles, CA: Diversity Program Consortium (DPC) Coordination and Evaluation Center at UCLA; 2020.

[15] ConronKJ, GoldbergSK. Adult LGBT population in the United States. 2019.

[16] GallupI. LGBT Identification in US Ticks Up to 7.1%. Retrieved 18 February 2022. 2022.

[17] HughesBE. Coming out in STEM: Factors affecting retention of sexual minority STEM students. Science advances. 2018;4(3):eaao6373. doi: 10.1126/sciadv.aao6373 29546240PMC5851677

[18] CechEA, WaidzunasTJ. Navigating the heteronormativity of engineering: The experiences of lesbian, gay, and bisexual students. Engineering Studies. 2011;3(1):1–24.

[19] CechEA, PhamMV. Queer in STEM organizations: Workplace disadvantages for LGBT employees in STEM related federal agencies. Social Sciences. 2017;6(1):12.10.3390/socsci6010012PMC1097804638550541

[20] Health NIo. NIH Workplace Climate and Harassment Survey Summary Findings Report. 2020.

[21] CarloneHB, JohnsonA. Understanding the science experiences of successful women of color: Science identity as an analytic lens. Journal of Research in Science Teaching: The Official Journal of the National Association for Research in Science Teaching. 2007;44(8):1187–218.

[22] TrujilloG, TannerKD. Considering the role of affect in learning: Monitoring students’ self-efficacy, sense of belonging, and science identity. CBE—Life Sciences Education. 2014;13(1):6–15. doi: 10.1187/cbe.13-12-0241 24591497PMC3940464

[23] MongelliF, PerroneD, BaLDUcciJ, SacchettiA, FerrariS, MatteiG, et al. Minority stress and mental health among LGBT populations: An update on the evidence. 2019.

[24] BrooksVR. Minority stress and lesbian women: Free Press; 1981.

[25] MeyerIH. Minority stress and mental health in gay men. Journal of health and social behavior. 1995:38–56. 7738327

[26] HurtadoS, AlvarezCL, Guillermo-WannC, CuellarM, ArellanoL. A model for diverse learning environments. Higher education: Handbook of theory and research: Springer; 2012. p. 41–122.

[27] CechE, WaidzunasT. Systemic inequalities for LGBTQ professionals in STEM. Science advances. 2021;7(3):eabe0933. doi: 10.1126/sciadv.abe0933 33523910PMC7810386

[28] MoyanoN, del Mar Sánchez-FuentesM. Homophobic bullying at schools: A systematic review of research, prevalence, school-related predictors and consequences. Aggression and violent behavior. 2020;53:101441.

[29] ElipeP, de la Oliva MuñozM, Del ReyR. Homophobic bullying and cyberbullying: Study of a silenced problem. Journal of homosexuality. 2018;65(5):672–86. doi: 10.1080/00918369.2017.1333809 28569622

[30] MustanskiB, MoskowitzD, MoranK, NewcombM, MacapagalK, Rodriguez-DiazC, et al. Evaluation of a stepped care eHealth HIV prevention program for diverse adolescent MSM: Protocol for a hybrid type 1 effectiveness-implementation trial of SMART (Preprint). JMIR Research Protocols. 2020;9. doi: 10.2196/19701 32779573PMC7448177

[31] MustanskiB. Ethical and regulatory issues with conducting sexuality research with LGBT adolescents: A call to action for a scientifically informed approach. Archives of sexual behavior. 2011;40(4):673–86. doi: 10.1007/s10508-011-9745-1 21528402

[32] RankinS, BlumenfeldW, WeberG, FrazerS. State of higher education for LGBT people: Campus pride 2010 national college climate survey. Charlotte, NC: Campus Pride. 2010.

[33] Mendoza-DentonR, DowneyG, PurdieVJ, DavisA, PietrzakJ. Sensitivity to status-based rejection: implications for African American students’ college experience. Journal of personality and social psychology. 2002;83(4):896. doi: 10.1037//0022-3514.83.4.896 12374443

[34] WorthingtonRL, NavarroRL, LoewyM, HartJ. Color-blind racial attitudes, social dominance orientation, racial-ethnic group membership and college students’ perceptions of campus climate. Journal of Diversity in higher education. 2008;1(1):8.

[35] ReisnerSL, ConronKJ, BakerK, HermanJL, LombardiE, GreytakEA, et al. “Counting” transgender and gender-nonconforming adults in health research: Recommendations from the gender identity in US surveillance group. Transgender Studies Quarterly. 2015;2(1):34–57.

[36] BenjaminiY, HochbergY. Controlling the False Discovery Rate: A Practical and Powerful Approach to Multiple Testing. Journal of the Royal Statistical Society: Series B (Methodological). 1995;57(1):289–300. 10.1111/j.2517-6161.1995.tb02031.x.

[37] FaulF, ErdfelderE, LangAG, BuchnerA. G*Power 3: a flexible statistical power analysis program for the social, behavioral, and biomedical sciences. Behav Res Methods. 2007;39(2):175–91. Epub 2007/08/19. doi: 10.3758/bf03193146 .17695343

[38] SadlerPM, SonnertG, HazariZ, TaiR. Stability and volatility of STEM career interest in high school: A gender study. Science Education. 2012;96(3):411–27. 10.1002/sce.21007.

[39] Education USDo. National Center for Education Statistics, Integrated Postsecondary Education Data System (IPEDS), Fall 2016 Completions Component. Digest of Education Statistics 2017; 2017.

[40] FeinsteinBA, DyarC. Bisexuality, minority stress, and health. Current sexual health reports. 2017;9(1):42–9. doi: 10.1007/s11930-017-0096-3 28943815PMC5603307

[41] MiritiMN. The elephant in the room: race and STEM diversity. BioScience. 2020;70(3):237–42.

[42] Allen-RamdialS-AA, CampbellAG. Reimagining the pipeline: Advancing STEM diversity, persistence, and success. BioScience. 2014;64(7):612–8. doi: 10.1093/biosci/biu076 25561747PMC4282132

[43] California Department of Education. Supporting LGBTQ+ Students. 2020.

[44] HallW. The effectiveness of policy interventions for school bullying: A systematic review. Journal of the Society for Social Work and Research. 2017;8(1):45–69. doi: 10.1086/690565 28344750PMC5363950

